The article "Studying the Effects of Cold Plasma Phosphorus Using Physiological and Digital Image Processing Techniques" was retracted in 2022. Reason: concerns about the peer review.

# Studying the Effects of Cold Plasma Phosphorus Using Physiological and Digital Image Processing Techniques

**DOI:** 10.1155/2022/8332737

**Published:** 2022-02-25

**Authors:** Malik Bader Alazzam, Walid Theib Mohammad, Mohammad Bani Younis, Ahmad Maher Al Sayeh, Fahima Hajjej, Ahmed S. AlGhamdi, Md Adnan Rahman

**Affiliations:** ^1^Faculty of Computer Science and Informatics, Amman Arab University, Jordan; ^2^Princess Aisha Bint Al Hussein College for Nursing and Health Sciences, Princess Aisha Nursing College, Al-Hussein Bin Talal University, Jordan; ^3^Department of Information Systems, College of Computer and Information Sciences, Princess Nourah bint Abdulrahman University, P.O. Box 84428, Riyadh 11671, Saudi Arabia; ^4^Department of Computer Engineering, Collage of Computers and Information Technology, Taif University, P.O. Box 11099, Taif 21944, Saudi Arabia; ^5^College of Business Administration (CBA), International University of Business Agriculture and Technology (IUBAT), Dhaka, Bangladesh

## Abstract

The goal of this study is to see how cold plasma affects rabbit bone tissue infected with osteoporosis. The search is divided into three categories: control, infected, and treated. The rabbits were subjected to cold plasma for five minutes in a room with a microwave plasma voltage of “175 V” and a gas flow of “2.” A histopathological photograph of infected bone cells is obtained to demonstrate the influence of plasma on infected bone cells, as well as the extent of destruction and effect of plasma therapy before and after exposure. The findings of the search show that plasma has a clear impact on Ca and vitamin D levels. In the cold plasma, the levels of osteocalcin and alkali phosphates (ALP) respond as well. Image processing techniques (second-order gray level matrix) with textural elements are employed as an extra proof. The outcome gives good treatment indicators, and the image processing result corresponds to the biological result.

## 1. Introduction

Many digital computer vision applications were developed in the early 1960s at Bell Laboratories [1], the Jet Engines Testing lab, the New England Technical University, the University of Maryland, and a few other research institutions, including satellite imagery, wire-photo specifications converting, diagnostic imaging, videoconferencing, character segmentation, and series of photos enhancement [2, 3]. The goal of early image processing was to boost the image's quality. It was created in order to improve people's visual effects. Image processing starts with a low-quality image and ends with a higher-quality image. Image enhancement, healing, coding, and compression are examples of image processing techniques. The American Jet Turbine Laboratory was the first to apply JPL. On the hundreds of lunar photographs collected by the Space Detector Ranger 7 in 1964, they employed image processing techniques such as template matching, gradation conversion, noise reduction, and others, taking into consideration the position of the sun and the moon's surroundings. The computer's ability to effectively map the moon's surface map is critical. Later, the spacecraft's over 100,000 images were subjected to more advanced image processing, resulting in the creation of a topographic map, colour map, and panoramic mosaic of the planet, which produced spectacular results and lay the groundwork for a human moon landing.

Processing was, nevertheless, rather expensive at the time, considering the status of computer technology. This began to change in the 1970s, when increasingly affordable computers and specialist equipment made digital imaging more accessible. In certain cases, such as television standard conversion, this resulted in photographs being processed in real time. As general-purpose computers evolved, they began to supplant specialist gear for all but the most specialized most computer-intensive applications. Digital pictures are presently the most frequent sort of image processing. Thanks to the availability of powerful computers and signal processors in the 2000s, it is extensively used since it is both the most adaptable and the most cost-effective method.

Plasma described as “electromagnetic energy in the GHz range” is known as microwave plasma. The animals used in the experiment showed no adverse effects [4–6]. The outcome of biological procedure employing the textural picture of the bone is proven using digital image processing. Textural qualities provide vital information about the tissue's surfaces and their interaction to one another [7–10]. Traditional textural qualities calculated using statistical features provide a textural feature known as the second-order matrix, which consists of four features that offer and produce information regarding textural decoration and structural elements. Any changes in the textural qualities employed as an indication for the alterations observed in the rabbit's bones are sensitive to these features [11].

Microwave plasma is a kind of plasma that is defined as having “electromagnetic energy in the GHz range.” The animals that were employed in the experiment exhibited no signs of illness. Digital image processing is used to verify the result of a biological method that makes use of the textural image of the bone as a guide.

Nonthermal plasma has several names in science. It is also known as gliding arc, plasma pencil, plasma needle, plasma jet, dielectric barrier discharge, and more (“one atmosphere uniform glow discharge plasma,” “atmospheric plasma,” “ambient pressure nonthermal discharges,” “nonequilibrium atmospheric pressure plasmas,” etc.). The NTP is nonthermal and operates at or near atmospheric pressure.

A tissue's textural properties give critical information regarding the surfaces of the tissue as well as their interaction with one another. Traditional textural qualities calculated using statistical features provide a textural feature known as the second-order matrix, which consists of four features that offer and produce information regarding textural decoration and structural elements. The second-order matrix is composed of four features that offer and produce information regarding textural decoration and structural elements. There is a strong relationship between these characteristics and any changes in textural qualities that are used as an indicator for the abnormalities detected in the rabbit's bones [12, 13].

## 2. Methodology

The rabbit samples (albino type) are collected according to sex and age, the rabbits are up to 3 months old, females are divided into three groups (control group, osteoporosis group, and plasma treatment group), and the laboratory procedure has been done as follows:

- Before inducing osteoporosis, collect 8 mL of blood via a cardiac puncture and separate the serum to determine vitamin D and calcium levels
- Cortisone medication 10 mg/daily for 7 weeks orally induced osteoporosis
- Take 8 mL of blood by heart puncture and separate serum to evaluate vitamin D and calcium levels after inducing osteoporosis in rabbits
- Give the sick rabbit's cold plasma for 9 minutes every day
-After treating with plasma, take 8 mL of blood by heart puncture and separate serum to assess vitamin D and calcium

The following are the laboratory methods:

1. The kit includes a working reagent; 1000 *μ*L from the working reagent has been mixed with 110 *μ*L from the sample and loading 255 in a well plate
2. The mixture is incubated at 38°C for 1 minute
3. Measure the change in absorbance per minute

(1) $$\begin{array}{c} \text{ALP Activity }\left(\text{U}/\text{L}\right)=\left(\text{OD}/\min.\right)\times 2750, \end{array}$$

where U/L indicates unit per liter.

### 2.1. Histological Analyses

The histology image of the bone was obtained in three cases: control, osteoporosis-infected, and plasma-treated; the gray level matrix was utilized to compute the textural characteristics; four features were calculated from this matrix; and the picture was transformed to gray scale to allow for analysis. The central pixel has been evaluated with its neighbors based on the size of window utilized to build the gray level matrix. The method is based on counting pixels that have the same texture characteristics that can occur in the picture [11].

Contrast is the difference in intensity between a pixel and its neighbor in a subimage; when the image is steady, the contrast is low, but in a variable intensity picture, the contrast is largest. The contrast equation is as follows [12, 14–20]:

(2) $$\begin{array}{c} C=\overset{\text{Ng}-1}{\underset{i=0}{\sum }}\overset{\text{Ng}-1}{\underset{j=0}{\sum }}{\left(i-j\right)}^{2}\;p\left(i,j\right), \end{array}$$

where *p*(*i*, *j*) is a histogram of a digital picture with intensity levels between [0, Ng-1], where Ng is the gray level value (0-255 or from 1 to 256).

Energy indicates the number of gray levels in the image, with a high energy value indicating a low number of gray levels and a low energy value indicating a large number of gray levels. The contrast equation is as follows [15]:

(3) $$\begin{array}{c} \text{Energy}=\overset{\text{Ng}-1}{\underset{i=0}{\sum }}\overset{\text{Ng}-1}{\underset{j=0}{\sum }}{\left[p\left(i,j\right)\right]}^{2}. \end{array}$$

The maximum value is one when the adjacent pixels are significantly connected and -1 when there are no relations. These characteristics are determined for the three instances: control, infected, and treated.

## 3. Main Results

In the control group, there are three rabbits that have not been treated. The second-order textural features contrast, correlation, energy, and homogeneity for trabecular bone and bone marrow are listed in Tables 1 and 2. Figures 1 and 2 show the control group's bone texture with a baseline picture and segmented one (trabecular bone and bone marrow).

In the infected group (osteoporosis), it includes 3 rabbits where doses of hydrocortisone and ovariectomy surgery were used to induce osteoporosis in the rabbits.  Figure 2 shows the bone texture for this group with the threshold image and segmentation (trabecular bone, bone marrow). Tables 1 and 2 list the second-order texture features contrast, correlation, energy, and homogeneity for trabecular bone tissue and bone marrow.

Figure 2 shows the texture histoimage, threshold, and segmentation for the infected group.

### 3.1. Cold Plasma Was Used to Treat the Group

It uses three rabbits, each of whom is treated with cold plasma for five minutes. Tables 1 and 2 state the second-order texture characteristics contrast, correlation, energy, and homogeneity for trabecular bone and bone marrow.  Figure 3 displays the skeletal texture for this group with a filter image and segmentation (trabecular bone, bone marrow).

The goal of the study was to see how cold plasma affected rabbit bones afflicted with osteoporosis, as well as to measure several biological characteristics (see Table 1). The findings of this table reveal that there has been a considerable shift in the Ca and vit which represents the statistic for the blood serum concentration. To declare that this value exhibits substantial modifications, the discrepancies between the calibration curve and the infected group with osteosarcoma value must be more than the least standard deviation value. The plasma-treated value is represented by the row in the table. The impact of plasma appears after a week of therapy, with the bones subject to five minutes each day. The *p* value indicates that there is a difference between the control, infected, and treated groups, while the significant value indicates that there is a difference between the three groups. In addition, the table shows that the control has the label, indicating that the values do not correspond, despite the fact that the bone is the same. The treated bones do not attain the same level of value as the control ones, but they are close. The average value for textural characteristics of trabecular bone tissue and bone marrow for the three groups is shown in Tables 1 and 2. Figures 2 and 4 depict the textural characteristics of trabecular bone tissue and bone marrow, respectively.

## 4. Conclusion

Elevated serum levels of alkaline phosphorus (ALP) suggest a problem in the bone, since this value increased in the infected group [4], and it was shown that there is a link between serum levels of osteocalcin and osteoporosis. It is true. According to some studies, high levels of osteocalcin in the blood are a sign of decreased bone density and a higher risk of fractures, so rabbits with high osteocalcin levels have weaker bones, which explains why bone reabsorption (the transition of minerals into the blood) discharges osteocalcin from the bone to the blood [5] and significantly lowers the levels of calcium and vitamin D in the blood serum because vitamin D deficiency in the serum of osteoporosis patients was linked to a decrease in calcium absorption because vitamin D is responsible for calcium absorption from the intestine and distribution to the body by regulating calcium distribution and blood deposition to the bone, and calcium is essential for bone mass building. It causes a reduction in the concentration of minerals in the bulk due to the bones and its thickness [6]. When infected samples were exposed to cold plasma, the cells in the skin absorbed it and converted it to protein vitamin D3, affecting skin and vitamin D production as well as metabolism to increase calcium absorption from the intestine and its calcification in the bone. As a result of this process, the levels of osteocalcin and ALP were reduced, as shown in Figures 1–3. The value of contrast in the infected group in the bone marrow is higher than that in the control and treated groups because the pixel intensity and neighbor intensity are very different in the infected group.  Figure 2 depicts the contrast, correlation, energy, and homogeneity values for trabecular bone tissue; the result reveals that the bone marrow responds to the plasma effect better than the trabecular bone.

## Figures and Tables

**Figure 1:** Trabecular bone of control.

**Figure 2:** Analysis for trabecular bone tissue of the infected group.

**Figure 3:** The texture histoimage, threshold, and segmentation for the treated group.

**Figure 4:** In the control, infected, and control groups, there is a substantial shift in Ca, vit D, osteocalcin, and ALP.

**Table 1:** The second-order texture analysis for trabecular bone of the control group.

No.	Contrast	Correlation	Energy	Homogeneity
1.	0.0522	0.77856	0.71564	0.88012
2.	0.05423	0.8976	0.52375	0.88132
3.	0.16425	0.67245	0.27343	0.8102
Average	0.074466	0.489466	0.46960	0.8572

**Table 2:** The second-order texture analysis for trabecular bone tissue of the infected group.

No.	Contrast	Correlation	Energy	Homogeneity
1.	0.10375	0.92395	0.46885	0.95025
2.	0.2752	0.94165	0.30605	0.9471
3.	0.114	0.9626	0.3286	0.95155
Average	0.164317	0.942733	0.367833	0.949633

## Data Availability

The data used to support the findings of this study are included within the article.
